# Research Progress of Deep Learning in the Diagnosis and Prevention of Stroke

**DOI:** 10.1155/2021/5213550

**Published:** 2021-08-09

**Authors:** Siqi Zhang, Miao Zhang, Shuai Ma, Qingyong Wang, Youyang Qu, Zhongren Sun, Tiansong Yang

**Affiliations:** ^1^Heilongjiang University of Chinese Medicine, No. 24 Heping Road, Harbin, China; ^2^Eighth Department of Acupuncture, Second Affiliated Hospital, Heilongjiang University of Chinese Medicine, Harbin 150001, China; ^3^Department of Neurology, The Second Affiliated Hospital of Harbin Medical University, No. 246 Xuefu Road, Harbin 150086, China; ^4^First Affiliated Hospital, Heilongjiang University of Chinese Medicine, No. 26 Heping Road, Harbin, China

## Abstract

In order to evaluate the importance of deep learning techniques in stroke diseases, this paper systematically reviews the relevant literature. Deep learning techniques have a significant impact on the diagnosis, treatment, and prediction of stroke. In addition, this study also discusses the current bottlenecks and the future development prospects of deep learning technology.

## 1. Stroke

Stroke (cerebral stroke), also known as “stroke,” “cerebrovascular accident” (cerebralvascular accident, CVA), is an acute cerebrovascular disease, characterized by high morbidity, high mortality, and high disability rate, accounting for 40% of the world's stroke deaths, the disability rate is as high as 70%, of which more than 40% of the severe disability [1], and the leading cause of death and disability accounting for about 12% of all deaths [2] poses a threat to human life health and work. In the acute stage of stroke, it is very important for clinicians to make accurate and rapid decisions, such as whether to use thrombolytic drugs or surgical intervention to preserve the damaged site. Medical imaging is the key method to diagnose ischemic stroke and the important basis for clinicians to choose treatment, where CT shows low density and DWI shows high signal that can identify ischemic tissue. Using these images, researchers can detect ischemic lesions and predict possible future lesions. At present, personal manual lesion tracking is still the gold standard for stroke lesion segmentation [3]. However, manual tracking takes a lot of time and labor, and even skilled operators take hours to mark. Therefore, how to objectively and accurately evaluate the information of ischemic stroke patients is a major challenge in clinical practice, which is particularly important for early warning of the high-risk population of ischemic stroke and reducing the incidence of stroke [4, 5]. The application of modern algorithms and data acquisition is particularly important. Diagnosis of early screening for ischemic stroke with deep learning [6] , automatic identification of the infarct size [7], and identification of vascular occlusion [8] all have better effect.

## 2. Deep Learning

Computer came out in the 1940s. With the development of more than 70 years, computer, as a new subject, not only involves natural science, computing, and other fields. In these only decades, computers have brought us progress in production and life. At the same time, human civilization has moved to a new level in the historical process. As the main function of the machine, the classical computing method includes decision tree, naive Bayes classification algorithm, random forest, *k*-means algorithm [9]. However, when we solve more and deeper practical problems, we find that traditional algorithms have many drawbacks. Artificial intelligence (artificial intelligence) was first proposed at the Dartmouth Conference in 1956 and belongs to the field of computer science [10]. The core of artificial intelligence is machine learning [11]. A mathematical method for simulating human neural network—deep learning—has been developed with the continuous upgrading and development of computer equipment. Malathi et al. [12] proposed mixed reasoning to predict disease and builds up *K*-nearest neighbor sum, fuzzy set theory, and case reasoning. The results show that this model can improve prediction accuracy. Shamdman et al. [13] developed a heart disease prediction system based on machine learning, a heart disease prediction system was developed. Through crossvalidation, the prediction accuracy of the SVM model was the highest. A team at Kyoto University in Japan used a deep neural network to read and translate human ideas, and “deep picture reconstruction” went beyond binary pixel information [14].

Recently, deep learning (DL, deep learning) has made outstanding contributions to industry and has been widely used in many other disciplines, especially in medical clinic to solve practical problems. It is a hot spot in the medical field. It uses multilayer artificial neural network (artificial neural network, ANN) to simulate the human brain [15]. The ANN is inspired by the CNS neural network, which consists of nodes connected together to form a network with variable weights between different connections. Just as countless neurons form our cerebral cortex, when humans perform daily functional activities, neurons release electrical signals to the central nervous system and other neurons, which people collect and apply various algorithms. Such as depth learning algorithm, these electrical signals are analyzed to guide the model construction. This is of great practical significance to realize artificial intelligence and deep analysis of brain working principle, leading machinery to “intelligence.”

## 3. Application of Depth Learning in Stroke Diagnosis

The division of the infarct size in early ischemic stroke is of great significance for the diagnosis and prediction of disease development. Stroke patients can determine the type of disease by CT, its price parity, noise impact that is small, and imaging speed that is better than other magnetic resonance imaging techniques [16, 17]. Then, there is the disadvantage of being unable to distinguish abnormal lesions. Magnetic resonance imaging can avoid this disadvantage, but it is expensive and inefficient [18]. Chen et al. [19] found that the DWI has the advantage of early diagnosis of acute ischemic stroke and can distinguish the boundary of new and old infarct, but due to time and technical constraints, it is difficult that MRI manually divide the early infarct volume. The Dice score of small lesions is 0.61 and that of large lesions is 0.83. The application of deep learning can mainly make diagnosis accurate and fully automatic. Yang [3] summarized the current segmentation methods and the development of deep neural network research and studies the depth learning-based segmentation methods for chronic or subacute stroke. A crosslayer fusion and contextual reasoning network (CLCI-Net) for T1-weighted images are proposed. Visual system and auxiliary analysis system are designed to reduce the pressure of clinician diagnosis and the error of subjective judgment. Acute ischemic stroke is difficult to detect in CT, and MRI perfusion images can detect key ischemic lesions; so, Chen [20] conducted the research of MRI data around stroke—MRI high precision segmentation of two-dimensional and three-dimensional fully convolutional neural networks—is based on level set [21], FCM based [22], and multiscale CNN [23].*D* sensitivity and accuracy of the *D* depth residual network are the highest compared with that of 3D cascaded non-symmetric residual U-Net. As an important part of stroke diagnosis, rehabilitation medicine has gradually moved towards intelligence, precision, and individuation, among which precision evaluation is the main direction. Lang [24] presents a series of automatic evaluation methods of the stroke upper limb motor function based on the depth learning system and puts forward a cyclic neural network model based on time attention for upper arm motion. Brunnstrom is the accuracy of expression by stages that can reach 100. The determination coefficient of the hand motor function score and clinician score can reach 0. A visual depth sensor was introduced to evaluate the function of the upper limb movement, which can track the position of upper limb bone space in real time. The agreement between automatic Fugl-Meyer score and clinician score was as high as 0.89. Image segmentation accuracy CT intracerebral hemorrhage is the basis of preventing early hematoma expansion in patients. However, there are many problems, such as blurred image edge, cavity phenomenon, and uneven gray scale. Wei [25], combining with the present, an algorithm model for image segmentation of cerebral hemorrhage CT based on curve evolution can automatically locate the hematoma suspected area profile, combining symbolic pressure functions with Letan polynomials, to improve the traditional calculation method. The above problems have been solved. Acute ischemic stroke (Als with large vessel occlusion,) with macrovascular occlusion Als-LVO) is one of the leading causes of stroke. Although intravenous thrombolysis is intravenous thrombosis, IVT is an effective way to treat Als, but the revascularization rate for the LVO of treatment is low. The curative effect is not good. Deep learning has been gradually applied to standardized LVO stroke diagnosis in recent years. Research shows that the sensitivity of CNN detection LVO is higher than that of the random forest algorithm (85% : 68%). Deep learning can improve the diagnosis rate of LVO stroke, increasing the speed of clinical work [26]. White matter hyperintense (white matter hyperintensity, WMH) is an imaging feature of diffuse small cerebral vascular disease and brain atrophy. WMH accurate segmentation of stroke lesions is related to the deep study of clinical medicine and epidemiology. WMH previous manual segmentation is very complicated, Guerrero, etc. [27] found that the convolution neural network can accurately distinguish the two lesions, and the CNN architecture is superior to other algorithms. The team of Mark and Mary Stevens Institute of Neuroimaging and Informatics (INI) at the University of Southern California, Stroke, said that they found an alternative, and this method allows clinicians to assess stroke damage without palliative injection of contrast media. Both magnetic resonance imaging and computed tomography require chemical contrast agents, and some contain high doses of X-radiation. Others may be harmful to patients with kidney or vascular disease. The depth learning algorithm designed by Wang Jiong's team can be derived from a safer type of the brain scan (pseudocontinuous artery spin-labeled magnetic resonance imaging, automatic extraction of stroke damage data in pCASL MRI). In the evaluation of brain damage in stroke patients, the pCASL deep learning model achieves 92% accuracy on both independent datasets and reduced damage during diagnosis [28].

## 4. Application of Depth Learning in Stroke Treatment

Collateral circulation can maintain the ability of brain tissue regeneration and is a determinant of the degree of recovery of ischemic stroke. Computer tomography (CTA) is widely used in the diagnosis of vascular diseases, which can provide important information of collateral circulation and is an important marker for evaluating collateral status. The application of deep learning function to the computer system can improve the ICC of consistency of CTA lateral branch cycle score from 0.58 to 0.77. Automatic CTA can provide objective collateral cycle score, which is highly consistent with expert CTA-CS and improves the reliability of CTA-CS. In conclusion [29], Ho et al. [30] use the method of deep learning, 118 cases of onset time were extracted to determine the specific onset time of patients. The combination of arterial spin labeling (ASL) and deep learning provides a more scientific treatment for acute ischemic stroke (AIS), which can better identify the low perfusion area. The area under the ROC is 0.958, which is better than the traditional algorithm [28]. TOAST classification is currently the most widely used stroke classification system, Ravi Garg included in 1091 patients with ischemic stroke, by comparing artificial TOAST and deep learning machine automatic TOAST, found that the two effects are close, and automatic classification can avoid the difference of artificial judgment to some extent, which is of guiding significance for the future analysis of the etiology and classification of ischemic stroke [31]. Rehabilitation exercise can help patients recover their daily functional, and exercise relearning is an essential process for stroke patients. The Chinese Guidelines for Early Rehabilitation of Stroke also include exercise rehabilitation as one of the core contents of stroke treatment [32]. However, modern rehabilitation has the disadvantages of high-cost and unsatisfactory effect [33]. The operation only requires the patient to cooperate with the rehabilitation therapist and complete the daily rehabilitation training under his guidance, but we know that low-level central nervous injury in stroke patients needs to induce nerve remodeling through active stimulation of motor nerves, which is the key to the rehabilitation of stroke patients. However, traditional rehabilitation therapy not only consumes manpower and material resources but also lacks the process of active shaping of patients. Hang [34] used depth learning technology and focusing on the recognition method of human action posture, an online rehabilitation action recognition model is established, which can realize the supervision and guidance of human action in the process of rehabilitation training. The action recognition equipment of rehabilitation training for wearing stroke is widely used in Ma Gaoyuan [35]. The recognition accuracy can be as high as 92.86.

## 5. Application of Depth Learning in Stroke Prediction

Deep learning also has a long-term contribution to stroke disease prediction. The prediction of ischemic stroke has a decision-making effect on its treatment. According to Heo et al. [29], a total of 2604 patients with acute ischemic stoke were included to estimate their mRS scores three months after onset. Three machine learning algorithms were used: deep neural networks, random forest, and rosette regression algorithms compared with the register (ASTRAL) scoring method for acute ischemic stroke in Lausanne, Switzerland. The deep neural network model outperformed the ASTRAL score, and there was no statistically significant difference between the performance and the ASTRAL score of the random forest and logical regression model. In accordance with Bacchi et al. [36], the application of deep learning to predict radiologic outcomes after thrombolytic therapy for acute ischemic stroke revealed an accuracy of 0.74 for both NIHSS24 score ≥ 4 and mRs90 score 0-1. Ma et al. [37]. It is found that the segmentation quality of ischemic stroke by depth learning tool is equal to or higher than that of manual segmentation, and the volume of ischemic core is highly consistent, which can provide reliable information for ischemic stroke prediction. In view of the lack of accuracy in assessing the risk rating of stroke patients in the current model, Yang et al. [38] designed the prediction model of stroke risk grade based on the maximum edge of the deep neural network can integrate stroke data with too large interclass divergence, improve the accuracy of prediction, and enhance clinical practicability. Yao et al. [39] in view of the design and construction of the prediction model system for cerebrovascular diseases, and based on the applicability of long-term and short-term memory (LSTM) neural network to the medical system, a disease prediction model LSTM neural network is proposed. The model is effective. Chen et al. [40] proposed a stroke prediction method characterized by deep learning and Mel frequency cepstrum coefficient (Mel Frequency Cestrum Coefficient, MFCC). The MFCC language features are trained in the convolution neural network model to obtain stroke prediction results. Experimental results show that the accuracy of test set and training set is higher than that of logistic regression. Recent studies have shown that convolutional neural networks are more suitable for medical imaging data [41]. Chauhan et al. have studied a deep learning approach based on convolutional neural networks that can predict the severity of language disorders by 3D lesions MRI by stroke patients.

## 6. Outlook

Nowadays, the aging of society is increasing day by day. Stroke, as the first leading cause of death in chronic diseases, has far exceeded the severity of cardiovascular disease and caused a serious burden on society and family. Today, advocating AI empowerment and AI to good, DL has involved many fields, such as words, numbers, and images, among which the medical field has outstanding contributions. Deep learning in the imaging study of ischemic stroke can accomplish intelligent segmentation, focus detection, image analysis, prediction, and treatment of ischemic stroke images by exploring deeper image information, so as to reduce human error and greatly improve the work efficiency of clinicians. Its development is deepening, which provides a more effective solution for the rehabilitation of patients in the future. The flexibility of the deep learning model also provides a more valuable tool for the study of multimodal combination.

Although deep learning research is becoming more and more mature, it can liberate the hands of clinicians to a certain extent, but the small sample size is still the biggest drawback, and there is no more clinical trials. Nat Med released a new guide to welcome artificial intelligence clinical research in 2020 [42], in order to further standardize the depth of learning in clinical promotion. In addition, the DL big data lacks the sharing way, and in the future, domestic hope establishes the more perfect database sharing platform. Of course, we should not ignore the importance of raw data and deep mining to find its pathological pathogenesis. Deep learning should be further blended with the morphology of ischemic stroke to lay the foundation for intelligence, comprehensive assessment of the pathogenesis of ischemic stroke, and early warning of disease occurrence.

A large number of deep learning research have been widely carried out, still facing more challenges. As a bridge and interdisciplinary subject between medical workers, the innovation and development of deep learning are the fundamental basis of this research, which is particularly important under the background of fierce international competition. Therefore, interdisciplinary indepth research is the source of artificial intelligence youth vitality, for personalized, accurate, modern medicine that laid the foundation. It is believed that with the emergence of more excellent experimental designs based on clinical efficacy, the deep excavation of deep learning will be further advanced.

## Data Availability

This article is a review article and does not contain relevant data.
